The article "Stability Analysis of an Extended SEIR COVID-19 Fractional Model with Vaccination Efficiency" was published in 2022. Journal: Comput Math Methods Med.

# Stability Analysis of an Extended SEIR COVID-19 Fractional Model with Vaccination Efficiency

**DOI:** 10.1155/2022/3754051

**Published:** 2022-09-20

**Authors:** Mubashara Wali, Sadia Arshad, Jianfei Huang

**Affiliations:** ^1^COMSATS University Islamabad, Lahore Campus, Pakistan; ^2^College of Mathematical Sciences, Yangzhou University, Yangzhou 225002, China

## Abstract

This work is aimed at presenting a new numerical scheme for *COVID-19* epidemic model based on Atangana-Baleanu fractional order derivative in Caputo sense (ABC) to investigate the vaccine efficiency. Our construction of the model is based on the classical SEIR, four compartmental models with an additional compartment V of vaccinated people extending it SEIRV model, for the transmission as well as an effort to cure this infectious disease. The point of disease-free equilibrium is calculated, and the stability analysis of the equilibrium point using the reproduction number is performed. The endemic equilibrium's existence and uniqueness are investigated. For the solution of the nonlinear system presented in the model at different fractional orders, a new numerical scheme based on modified Simpson's 1/3 method is developed. Convergence and stability of the numerical scheme are thoroughly analyzed. We attempted to develop an epidemiological model presenting the *COVID-19* dynamics in Italy. The proposed model's dynamics are graphically interpreted to observe the effect of vaccination by altering the vaccination rate.

## 1. Introduction

Emerging in December 2019, *COVID-19* became the biggest global threat. The whole world faced a critical situation, and a panic was created throughout the globe. The World Health Organization (WHO) declared it as an international health emergency. Not much was known about this virus as it was a new virus that has not been identified earlier in humans. So, relying on the observations and symptoms shown by the people who caught the virus, strategies of isolation, lockdown, and social distancing were adopted to prevent the disease from spreading. With the passage of time, the virus becomes more threatening because of its new variants. To investigate the dynamics and transmission of the virus, researchers utilized the concept of mathematical modeling [1–4]. These models actually do not provide the cure for the infectious diseases but can contribute in predicting the dynamics and behaviour of these infections through simulations.

Researchers rely more on fractional models because of their nonlocal behaviour, hereditary properties, and memory effects rather than integer order models. Besides, a number of experimental facts exhibit that the natural dynamics go along with fractional calculus. Ahmad et al. [5] utilized the modified Euler's method to study the dynamics of the model for *COVID-19* based on fractional differential equations and simulate the results by using the available data of initial days of the spread in Wuhan City. Zakary et al. [6] investigated the situation of the spread of the Corona Virus under the effect of two classes, quarantined and other who did not respect the quarantine strategy using the mathematical model, and an optimal control strategy to reduce the infections in Morocco. Ahmad et al. [7] presented a brief analysis on the WHO reported data for Pakistan and investigated it using the SEIR fractional model. Askar et al. [8] considered the SITR fractional model to forecast the transmission of deadly virus along with imposed lockdown in India. Bushnaq et al. [9] investigated the effect of physical distance to control the spread of the virus through fractional order model. Abdulwasaa et al. [10] proposed a fractal fractional model for forecasting deaths and new cases of *COVID-19* outbreak in India. Baba and Rihan [11] used the Caputo-Fabrizio fractional order model to analyze the dynamics of *COVID-19* variants. A fractional order delay differential model for *COVID-19* infection was provided by Rihan and Gandhi [12] to understand what triggers the severity of symptoms and disease of polluted lung and respiratory system. A stochastic SIAQR epidemic model was proposed by Rihan and Alsakaji [13] to understand the dynamics of *COVID-19*. Furati et al. [14] tested the data taken from China, Saudi Arabia, Brazil, and Italy by proposing a numerical scheme using fractional order model performing the two-step generalized exponential time-differencing method. Alqahtani [15] numerically analyzed and investigated the stability of the SIR epidemic model considering the health system. Recently another fractional order derivative with nonsingular kernel named as Generalized Hattaf Fractional (GHF) derivative [16] is introduced. We can see the use of this derivative for epidemiological models in recent literature. By creating a new numerical method, Hattaf [17] investigated the qualitative properties of solutions to fractional differential equations with the new GHFs derivative, including stability, asymptotic stability, and Mittag-Leffler stability and later applied the obtained analytical and numerical results to a biological nonlinear system derived from epidemiology. Cheneke et al. [18] developed and examined a coinfection of HIV and cholera model using GHF derivative and the solution's behaviour is deciphered. In present work we have used ABC derivative for our proposed model. However, we can extend our work using the GHF derivative for fractional order mathematical models in future.

Despite all the measures taken to control the virus, *COVID-19* remained a threat because of its high propagation rate leaving the majority of the population susceptible to the disease and escalating the need to develop a suitable and effective vaccine. The process to gain immunity against *COVID-19* is still under discussion. Most of the people infected with *COVID-19* developed the immunity against the virus, but still it is unknown how long this immunity will last as there are some reported cases of getting the infection for a second time. In this situation, the only solution to gain herd immunity is mass vaccination. Hence, to achieve this milestone, vaccination is required for a huge portion of the global population. In this regard, WHO helped governments to launch and refine their vaccination programmes along with UNICEF, Gavi, and partners. According to reference [19], 43.5% of the world population has been given at least one shot of *COVID-19* vaccine till the 21^st^ of September 2021. Modified mathematical models with an additional compartment of the vaccinated class are discussed in recent literature to foresee the efficacy, effect, and dynamics of the vaccination. Meng et al. [20] established an SEIRV model to differentiate between the effects of mandatory and voluntary vaccination methods on heterogeneous networks. Ramos et al. [21] investigated the impact of variants and vaccines on the spread of *COVID-19* applying the model to Italy as a test case. Tetteh et al. [22] analyzed the mass and ring vaccination strategies to control the transmission of SARS-CoV-2 by varying vaccine efficacy rate. Harizi et al. [23] used the SIRV model to check the future dynamics of the pandemic by varying vaccination rates in Canada. Karabay et al. [24] presented an SEIR simulator to model effective immunization and sterilizing outcomes in order to assess the vaccination effect. Tuteja [25] numerically solved the modified SEIR model including the vaccinated class to investigate the viral dynamics of the epidemic. Ghostine [26] proposed an SEIR model with an extension of the vaccination compartment to investigate the effect of vaccination in Saudi Arabia. Wintachaia and Prathomb [27] presented a detailed stability analysis of the *COVID-19* epidemic model to investigate the vaccine efficiency. Alsakaji et al. [28] examined the dynamics of *COVID-19* in the UAE using an exptended SEIR epidemic model with vaccination, temporal delays, and random noise. For transmission of the infectious disease, Kou et al. [29] established a multiscale agent-based model to investigate the impact of nonpharmaceutical interventions and vaccination. Acuña-Zegarra. [30] formulated a *COVID-19* optimal control problem to study the efficacy and responses of the vaccine induced immunity. Albani et al. [31] estimated the parameters of SEIR like epidemic model using daily reports of *COVID-19* of New York and Chicago to analyze the impact caused by vaccination delay.

Motivated from the above studies, we have presented in this work a modified SEIRV epidemic model with an additional compartment of vaccinated individuals to examine the effectiveness and efficacy of the vaccine by varying its rate considering the ABC derivative. We have used ABC fractional order derivative because a number of experimental facts exhibit that the natural dynamics go along with fractional calculus as the fractional order derivatives are nonlocal in behaviour and possess the hereditary properties and memory effects. Also, we have constructed a new, more efficient, and effective numerical scheme for fractional differential equation with Atangana-Baleanu derivative in Caputo sense using Simpson's 1/3 method for the approximation of the integral function involved in the problem.

The paper comprises different sections. In section 2, some basic definitions are recalled which have been used in the work later. SEIRV epidemic model for *COVID-19* is presented in section 3. The equilibrium points and the basic reproduction number using next generation method are calculated, and the stability of these points is also analyzed in this section. For the solution of the proposed model modified Simpson's 1/3 method alongside complete stability and convergence analysis, it is presented in section 4. Conversion of mathematical model to fractional order model is given in section 5. Numerical simulations are also presented in the same section.

## 2. Preliminaries

This part will review some of the fundamental definitions of fractional calculus, which will be useful in the subsequent work.

**Definition 1 .**

For *x* ∈ *ℍ*^1^(0, *T*) and 0 < *ϑ* < 1, the *ϑ*th–order ABC derivative and integral of *x*(*t*) are defined [32] as

(1) $$\begin{array}{c} {\;}^{\text{ABC}}D^{\vartheta }x\left(t\right)≔\frac{J\left(\vartheta \right)}{1-\vartheta }\int_{0}^{t}E_{\vartheta }\left[-\frac{\vartheta }{1-\vartheta }{\left(t-\xi \right)}^{\vartheta }\right]\dot{x}\left(\xi \right)d\xi , \end{array}$$

(2) $$\begin{array}{c} {\;}^{\text{ABC}}I^{\vartheta }x\left(t\right)≔\frac{1-\vartheta }{J\left(\vartheta \right)}x\left(t\right)+\frac{\vartheta }{J\left(\vartheta \right)\Gamma \left(\vartheta \right)}\int_{0}^{t}{\left(t-\xi \right)}^{\vartheta -1}x\left(\xi \right)d\xi , \end{array}$$

where *J*(*ϑ*) represents the normalization function given by

(3) $$\begin{array}{c} J\left(\vartheta \right)=1-\vartheta +\frac{\vartheta }{\Gamma \left(\vartheta \right)}, \end{array}$$

with *J*(*ϑ*)|_*ϑ*=0,1_ = 1 and *E*_*ϑ*_ is the Mittag-Leffler function defined as *E*_*ϑ*_(*z*) = ∑_*n*=0_^∞^(*z*^*n*^/Γ(*nϑ* + 1)).

The lemma below presents the Gronwall inequality [33], which will be used for the proof of our main result.

**Lemma 1 .**

The Gronwall inequality for fractional order differential equation states

Let *C*_1_ > 0 independent of *δt*, *C*_2_ ≥ 0 and {*u*_*n*_} satisfy the inequality

(4) $$\begin{array}{c} \left|u_{n}\right|\leq {\left(\delta t\right)}^{\vartheta }C_{1}\overset{n-1}{\underset{l=0}{\sum }}{\left(n-l\right)}^{\vartheta -1}\left|u_{j}\right|+C_{2},l=0,1,\cdots ,n-1,n\delta t\leq T, \end{array}$$

with 0 < *ϑ* ≤ 1. Then

(5) $$\begin{array}{c} \left|u_{n}\right|\leq C_{2}E_{\vartheta }\left(C_{1}\Gamma \left(\vartheta \right)T^{\vartheta }\right),n\delta t\leq T, \end{array}$$

where the parameter *E*_*ϑ*_ is the Mittage-Leffler function. Particularly when *ϑ* = 1, inequality (5) becomes

(6) $$\begin{array}{c} \left|u_{n}\right|\leq C_{2}e^{C_{1}T},n\delta t\leq T. \end{array}$$

In this study, we used an SEIR model with vaccination effectiveness to forecast the COVID-19 condition when a vaccine is released.

## 3. Mathematical Model

Mathematical models are of great importance in predicting the behaviour of the viral epidemic diseases. There are a number of models which can be used to describe and investigate the spread of the disease. Recently *COVID-19* emerged as a viral epidemic, and we are not aware enough about the behaviour and spread of this virus. To investigate the *COVID-19* situation under the effect of vaccination, we consider the following SEIRV epidemic disease model:

(7) $$\begin{array}{c} \dot{S}=\Lambda -\mu S-\delta S-\beta S\frac{I}{N},\\ \dot{E}=\beta S\frac{I}{N}-\left(\mu +\varepsilon \right)E+\sigma \beta V\frac{I}{N},\\ \dot{I}=\varepsilon E-\left(\gamma +\mu +\rho \right)I,\\ \dot{R}=\gamma I-\mu R,\\ \dot{V}=\delta S-\mu V-\sigma \beta V\frac{I}{N}. \end{array}$$

To define the model equations, the total population, represented by *N*, is separated into susceptible, exposed, infected, recovered, and vaccinated classes denoted by *S*(*t*), *E*(*t*), *I*(*t*), *R*(*t*), and *V*(*t*). The flow chart of the above system is shown in Figure 1.

The above system of equation (7) is subject to the initial conditions

(8) $$\begin{array}{c} S\left(0\right)=S_{0},E\left(0\right)=E_{0},I\left(0\right)=I_{0},R\left(0\right)=R_{0},V\left(0\right)=V_{0}, \end{array}$$

and the following are the parameters:

*μ*: per-capita natural death rate,

*γ*: the rate at which infectious people recover,

*ρ*: average fatality rate for virus-infected people,

*β*: disease transmission probability per contact times the amount of contacts made per unit of time (dimensionless),

*Λ*: the birth rate per-capita,

*ε*: progression rate from E to I,

1/*γ*: contagious period,

1/*ε*: incubation period,

*δ*: vaccination rate,

*σ*: vaccine ineffectiveness, 0 ≤ *σ* ≤ 1, 

1 − *σ*: vaccine effectiveness,

having T units per unit of time.

### 3.1. Stability Analysis of SEIRV *COVID-19* Model

In this section, stability analysis will be carried out to find the disease-free equilibrium and endemic equilibrium points. In order to get these points, each of the equations given in system of equation (7) will be equated to zero.

### 3.2. Disease-Free Equilibrium and the Basic Reproduction Number (**R**_0_)

Because there is no disease propagation in disease-free equilibrium, so *I* = 0, and hence we get

(9) $$\begin{array}{c} S^{0}=\frac{\Lambda }{\mu +\delta },\\ E^{0}=0,R^{0}=0,\\ V^{0}=\frac{\delta \Lambda }{\mu \left(\mu +\delta \right)}, \end{array}$$

so the disease-free equilibrium point is *𝔼*^0^(*S*^0^, *E*^0^, *I*^0^, *R*^0^, *V*^0^) = (*Λ*/(*μ* + *δ*), 0, 0, 0, *δΛ*/*μ*(*μ* + *δ*)).

The average number of secondary infections induced by an infectious individual is given by the basic reproduction number *R*_0_. It estimates the growth of the virus outbreak. The basic reproduction number *R*_0_ is determined using the next generation method [34]. Using $\dot{E}$ and $\dot{I}$ from system of equation (7), the Jacobian matrices of the disease-free equilibrium are as follows:

(10) $$\begin{array}{c} F=\left[\begin{array}{cc} 0 & \beta S^{0}+\sigma \beta V^{0}\\ 0 & 0 \end{array}\right],U=\left[\begin{array}{cc} \mu +\varepsilon & 0\\ -\varepsilon & \gamma +\mu +\rho \end{array}\right],\\ U^{-1}=\frac{1}{\left(\mu +\varepsilon \right)\left(\gamma +\mu +\rho \right)}\left[\begin{array}{cc} \gamma +\mu +\rho & 0\\ \varepsilon & \mu +\varepsilon \end{array}\right],\\ FU^{-1}=\frac{1}{\left(\mu +\varepsilon \right)\left(\gamma +\mu +\rho \right)}\left[\begin{array}{cc} 0 & \beta S^{0}+\sigma \beta V^{0}\\ 0 & 0 \end{array}\right]\left[\begin{array}{cc} \gamma +\mu +\rho & 0\\ \varepsilon & \mu +\varepsilon \end{array}\right],\\ FU^{-1}=\frac{1}{\left(\mu +\varepsilon \right)\left(\gamma +\mu +\rho \right)}\left[\begin{array}{cc} \beta \varepsilon S^{0}+\sigma \beta \varepsilon V^{0} & \left(\beta S^{0}+\sigma \beta V^{0}\right)\left(\mu +\varepsilon \right)\\ 0 & 0 \end{array}\right]. \end{array}$$

Here *FU*^−1^ is the next generation matrix and we can obtain the basic reproduction number as *R*_0_ = *ρ*(*FU*^−1^), so

(11) $$\begin{array}{c} R_{0}=\frac{\left(\beta \varepsilon S^{0}+\beta \varepsilon \sigma V^{0}\right)}{\left(\mu +\varepsilon \right)\left(\gamma +\mu +\rho \right)}. \end{array}$$

Substituting the values of *S*^0^ and *V*^0^, the following value of the reproduction number is obtained for the system of equation (7):

(12) $$\begin{array}{c} R_{0}=\frac{\beta \varepsilon \Lambda \left(\mu +\delta \sigma \right)}{\mu \left(\mu +\delta \right)\left(\mu +\varepsilon \right)\left(\gamma +\mu +\rho \right)}. \end{array}$$

**Theorem 1 .**

If *R*_0_ < 1 then the *COVID-19* model of equation (7) disease-free equilibrium point is locally asymptotically stable.

**Proof**

The Jacobian of system of equation (7) is given as

(13) $$\begin{array}{c} J=\left[\begin{array}{ccccc} -\mu -\delta -\frac{\beta I}{N} & 0 & -\frac{\beta S}{N} & 0 & 0\\ \frac{\beta I}{N} & -\left(\mu +\varepsilon \right) & \frac{\beta S}{N}+\frac{\sigma \beta V}{N} & 0 & \frac{\sigma \beta I}{N}\\ 0 & \varepsilon & -\left(\gamma +\mu +\rho \right) & 0 & 0\\ 0 & 0 & \gamma & -\mu & 0\\ \delta & 0 & -\frac{\sigma \beta V}{N} & 0 & -\mu \end{array}\right]. \end{array}$$

Jacobian around disease-free equilibrium point *𝔼*^0^((*Λ*/*μ* + *δ*), 0, 0, 0, (*δΛ*/*μ*(*μ* + *δ*))) is

(14) $$\begin{array}{c} J^{0}=\left[\begin{array}{ccccc} -\mu -\delta & 0 & -\frac{\beta \Lambda }{\mu +\delta } & 0 & 0\\ 0 & -\left(\mu +\varepsilon \right) & \frac{\beta \Lambda }{\mu +\delta }+\frac{\sigma \beta \delta \Lambda }{\mu \left(\mu +\delta \right)} & 0 & 0\\ 0 & \varepsilon & -\left(\gamma +\mu +\rho \right) & 0 & 0\\ 0 & 0 & \gamma & -\mu & 0\\ \delta & 0 & -\frac{\sigma \beta \delta \Lambda }{\mu \left(\mu +\delta \right)} & 0 & -\mu \end{array}\right]. \end{array}$$

We can observe from the preceding matrix that three of its eigenvalues *λ*_1,2_ = −*μ*, *λ*_3_ = −*μ* − *δ* are negative and we are left with

(15) $$\begin{array}{c} J^{0}=\left[\begin{array}{cc} -\left(\mu +\varepsilon \right) & \frac{\beta \Lambda }{\mu +\delta }+\frac{\sigma \beta \delta \Lambda }{\mu \left(\mu +\delta \right)}\\ \varepsilon & -\left(\gamma +\mu +\rho \right) \end{array}\right]. \end{array}$$

Now from above matrix, the last two eigenvalues are

(16) $$\begin{array}{c} \lambda_{4}=-\frac{1}{2}\left(\varpi_{1}+\varpi_{2}+\sqrt{{\left(\varpi_{1}-\varpi_{2}\right)}^{2}+4\varpi_{1}\varpi_{2}R_{0}}\right),\\ \lambda_{5}=-\frac{1}{2}\left(\varpi_{1}+\varpi_{2}-\sqrt{{\left(\varpi_{1}-\varpi_{2}\right)}^{2}+4\varpi_{1}\varpi_{2}R_{0}}\right), \end{array}$$

where *ϖ*_1_ = (*μ* + *ε*) and *ϖ*_2_ = (*γ* + *μ* + *ρ*), and for *R*_0_ < 1, we have *λ*_4_ < 0 and *λ*_5_ < 0.

Hence for *R*_0_ < 1 the disease-free equilibrium is locally asymptotically stable.

### 3.3. Existence and Uniqueness of Endemic Equilibrium

In order to investigate the existence and uniqueness of the endemic equilibrium *𝔼*^∗^ for *R*_0_ > 1, we will set all the derivatives of model of equation (7) equals to zero. Let *𝔼*^∗^ = (*S*^∗^, *E*^∗^, *I*^∗^, *R*^∗^, *V*^∗^) be the endemic equilibrium of model of equation (7). Then by solving the following equations we can obtain the endemic equilibrium.

(17) $$\begin{array}{c} \Lambda -\mu S^{*}-\delta S^{*}-\beta S^{*}\frac{I^{*}}{N}=0,\\ \beta S^{*}\frac{I^{*}}{N}-\left(\mu +\varepsilon \right)E^{*}+\sigma \beta V^{*}\frac{I^{*}}{N}=0,\\ \varepsilon E^{*}-\left(\gamma +\mu +\rho \right)I^{*}=0,\\ \gamma I^{*}-\mu R^{*}=0,\\ \delta S^{*}-\mu V^{*}-\sigma \beta V^{*}\frac{I^{*}}{N}=0. \end{array}$$

Now, solving first, third, and fourth equations of equation (17), we get

(18) $$\begin{array}{c} S^{*}=\left(\frac{\Lambda }{\mu +\delta +\left(\beta I^{*}/N\right)}\right),E^{*}=\left(\frac{\gamma +\mu +\rho }{\varepsilon }\right)I^{*},R^{*}=\left(\frac{\gamma }{\mu }\right)I^{*}. \end{array}$$

Also equation (17) gives

(19) $$\begin{array}{c} V^{*}=\frac{\beta S^{*}I^{*}}{\mu N}-\frac{\left(\mu +\varepsilon \right)}{\mu }E^{*}+\frac{\delta }{\mu }S^{*}. \end{array}$$

The following quadratic equation for *I*^∗^ is obtained:

(20) $$\begin{array}{c} A{\left(I^{*}\right)}^{2}+BI^{*}+C=0, \end{array}$$

where

(21) $$\begin{array}{c} A=\sigma \beta^{2\rho }\left(\mu +\varepsilon \right)\left(\gamma +\mu +\rho \right),\\ B=\mu N\left(\mu +\varepsilon \right)\left(\gamma +\mu +\rho \right)\beta +\sigma \beta \left(\mu +\varepsilon \right)\left(\gamma +\mu +\rho \right)N-N\sigma \Lambda \beta^{2\rho }\varepsilon ,\\ C=\mu N^{2}\left(\mu +\delta \right)\left(\mu +\varepsilon \right)\left(\gamma +\mu +\rho \right)\left(1-R_{0}\right). \end{array}$$

It is evident that *A* is always positive while *C* is negative for *R*_0_ > 1. Hence, there exists a positive and unique value of *I*^∗^, which results in a unique endemic equilibrium for *R*_0_ > 1.

## 4. Numerical Approximation

Consider the nonlinear fractional order differential equation

(22) $$\begin{array}{c} \begin{array}{c} {}^{\text{ABC}}D^{\vartheta }x\left(\tau \right)=f\left(x\left(\tau \right),\tau \right),0<\tau <T<\infty ,\\ x=\left(0\right)=x_{0}, \end{array} \end{array}$$

where 0 < *ϑ* < 1. The vector function *f* in the differential equation is real valued and continuous and satisfies the Lipschitz condition.

(23) $$\begin{array}{c} \left\|f\left(x_{1}\left(\tau \right)\right)-f\left(x_{2}\left(\tau \right)\right)\right\|\leq L\left\|x_{1}\left(\tau \right)-x_{2}\left(\tau \right)\right\|,L>0. \end{array}$$

To derive the numerical scheme for the above mentioned nonlinear fractional order differential equation, the given interval [0, *T*] will be subdivided into equal intervals with time step *δτ* = *T*/*N*, where *δτ*_*n*+1_ − *δτ*_*n*_ = *δτ* for *n* = 0, 1, 2, ⋯, *N* − 1. For convenience, the approximate solution of *x*(*τ*_*n*_) will be denoted by *x*_*n*_ with *δτ*_*n*_ = *nδτ*, *n* = 0, 1, 2, ⋯, *N*.

Applying the integral operator of equation (2) on equation (22), we get

(24) $$\begin{array}{c} x\left(\tau \right)=x_{0}+I^{\vartheta }f\left(x\left(\tau \right),\tau \right),0<\tau <T<\infty , \end{array}$$

where the integral *I*^*ϑ*^ in the above equation is the ABC integral. Using equation (2) to discretize the integral *I*^*ϑ*^, we get

(25) $$\begin{array}{c} {\;}^{\text{ABC}}I^{\vartheta }f\left(x\left(\tau_{n+1}\right),\tau_{n+1}\right)=\frac{\left(1-\vartheta \right)}{J\left(\vartheta \right)}f\left(x\left(\tau_{n+1}\right),\tau_{n+1}\right)+\frac{\vartheta }{J\left(\vartheta \right)\Gamma \left(\vartheta \right)}\int_{0}^{\tau_{n+1}}{\left(\tau_{n+1}-s\right)}^{\vartheta -1}f\left(x\left(s\right),s\right)ds,n=0,1,2,\cdots ,N-1. \end{array}$$

*f*(*x*(*s*)) is approximated on each subinterval [*τ*_*i*_, *τ*_*i*+1_], by the following piecewise quadratic interpolation polynomial.

(26) $$\begin{array}{c} {\left.f\left(x\left(s\right),s\right)\right|}_{\tau_{i},\tau_{i+1}}\approx \frac{\left(\tau_{i+1}-s\right)\left(\tau_{i+1/2}-s\right)}{\left(\tau_{i}-\tau_{i+1}\right)\left(\tau_{i}-\tau_{i+1/2}\right)}f\left(x\left(\tau_{i}\right),\tau_{i}\right)+\frac{\left(\tau_{i+1}-s\right)\left(\tau_{i}-s\right)}{\left(\tau_{i+1/2}-\tau_{i+1}\right)\left(\tau_{i+1/2}-\tau_{i}\right)}f\left(x\left(\tau_{i+1/2}\right),\tau_{i+1/2}\right)+\frac{\left(\tau_{i+1/2}-s\right)\left(\tau_{i}-s\right)}{\left(\tau_{i+1}-\tau_{i}\right)\left(\tau_{i+1}-\tau_{i+1/2}\right)}f\left(x\left(\tau_{i+1}\right),\tau_{i+1}\right), \end{array}$$

where *τ*_*i*+1/2_ = (*τ*_*i*_ + *τ*_*i*+1_)/2 is mid point of the interval [*τ*_*i*_, *τ*_*i*+1_].

Also, the value of *f*(*x*(*τ*_*i*+1/2_), *τ*_*i*+1/2_) will be approximated using the interpolation

(27) $$\begin{array}{c} f\left(x\left(\tau_{i+1/2}\right),\tau_{i+1/2}\right)=\frac{1}{2}f\left(x\left(\tau_{i}\right),\tau_{i}\right)+\frac{1}{2}f\left(x\left(\tau_{i+1}\right),\tau_{i+1}\right). \end{array}$$

Putting equation (27) in equation (26), we get

(28) $$\begin{array}{c} {\left.f\left(x\left(s\right),s\right)\right|}_{\tau_{i},\tau_{i+1}}\approx \frac{\left(\tau_{i+1}-s\right)\left(\tau_{i+1/2}-s\right)}{\left(\tau_{i}-\tau_{i+1}\right)\left(\tau_{i}-\tau_{i+1/2}\right)}f\left(x\left(\tau_{i}\right),\tau_{i}\right)+\frac{\left(\tau_{i+1}-s\right)\left(\tau_{i}-s\right)}{\left(\tau_{i+1/2}-\tau_{i+1}\right)\left(\tau_{i+1/2}-\tau_{i}\right)}\left(\frac{1}{2}f\left(x\left(\tau_{i}\right),\tau_{i}\right)+\frac{1}{2}f\left(x\left(\tau_{i+1}\right),\tau_{i+1}\right)\right)+\frac{\left(\tau_{i+1/2}-s\right)\left(\tau_{i}-s\right)}{\left(\tau_{i+1}-\tau_{i}\right)\left(\tau_{i+1}-\tau_{i+1/2}\right)}f\left(x\left(\tau_{i+1}\right),\tau_{i+1}\right)\\ =\frac{2}{{\left(\delta \tau \right)}^{2}}\left(\left(\left(\tau_{i+1}-s\right)\left(\tau_{i+1/2}-s\right)-\left(\tau_{i+1}-s\right)\left(\tau_{i}-s\right)\right)f\left(x\left(\tau_{i}\right),\tau_{i}\right)+\left(\left(\tau_{i+1/2}-s\right)\left(\tau_{i}-s\right)-\left(\tau_{i+1}-s\right)\left(\tau_{i}-s\right)\right)f\left(x\left(\tau_{i+1}\right),\tau_{i+1}\right)\right). \end{array}$$

Using above approximation, equation (25) takes the form

(29) $$\begin{array}{c} {}^{\text{ABC}}I^{\vartheta }f\left(x\left(\tau_{n+1}\right),\tau_{n+1}\right)=\frac{\left(1-\vartheta \right)}{J\left(\vartheta \right)}f\left(x\left(\tau_{n+1}\right),\tau_{n+1}\right)+\frac{\vartheta }{J\left(\vartheta \right)}\frac{2}{{\left(\delta \tau \right)}^{2}\Gamma \left(\vartheta \right)}\overset{n}{\underset{i=0}{\sum }}\left(\int_{\tau_{i}}^{\tau_{i+1}}{\left(\tau_{n+1}-s\right)}^{\vartheta -1}\left(\left(\left(\tau_{i+1}-s\right)\left(\tau_{i+1/2}-s\right)-\left(\tau_{i+1}-s\right)\left(\tau_{i}-s\right)\right)f\left(x\left(\tau_{i}\right),\tau_{i}\right)+\left(\left(\tau_{i+1/2}-s\right)\left(\tau_{i}-s\right)-\left(\tau_{i+1}-s\right)\left(\tau_{i}-s\right)\right)f\left(x\left(\tau_{i+1}\right),\tau_{i+1}\right)\right)\right) \end{array}$$

(30) $$\begin{array}{c} =\frac{\left(1-\vartheta \right)}{J\left(\vartheta \right)}f\left(x\left(\tau_{n+1}\right),\tau_{n+1}\right)+\frac{\vartheta }{J\left(\vartheta \right)}\frac{2}{{\left(\delta \tau \right)}^{2}\Gamma \left(\vartheta \right)}\left[\int_{\tau_{0}}^{\tau_{1}}{\left(\tau_{n+1}-s\right)}^{\vartheta -1}\left(\left(\tau_{1}-s\right)\left(\tau_{1/2}-s\right)-\left(\tau_{1}-s\right)\left(\tau_{0}-s\right)\right)f\left(x\left(\tau_{0}\right),\tau_{0}\right)ds+\int_{\tau_{0}}^{\tau_{1}}{\left(\tau_{n+1}-s\right)}^{\vartheta -1}\left(\left(\tau_{0}-s\right)\left(\tau_{1/2}-s\right)-\left(\tau_{1}-s\right)\left(\tau_{0}-s\right)\right)f\left(x\left(\tau_{1}\right),\tau_{1}\right)ds+\overset{n-1}{\underset{k=1}{\sum }}\int_{\tau_{i}}^{\tau_{i+1}}{\left(\tau_{n+1}-s\right)}^{\vartheta -1}\left(\left(\left(\tau_{i+1}-s\right)\left(\tau_{i+1/2}-s\right)-\left(\tau_{i+1}-s\right)\left(\tau_{i}-s\right)\right)f\left(x\left(\tau_{i}\right),\tau_{i}\right)\right.\left.+\left(\left(\tau_{i}-s\right)\left(\tau_{i+1/2}-s\right)-\left(\tau_{i+1}-s\right)\left(\tau_{i}-s\right)\right)f\left(x\left(\tau_{i+1}\right),\tau_{i+1}\right)\right)ds+\int_{t_{n}}^{\tau_{n+1}}{\left(\tau_{n+1}-s\right)}^{\vartheta -1}\left(\left(\tau_{n+1}-s\right)\left(\tau_{n+1/2}-s\right)-\left(\tau_{n+1}-s\right)\left(t_{n}-s\right)\right)f\left(x\left(\tau_{n}\right),\tau_{n}\right)ds+\int_{t_{n}}^{\tau_{n+1}}{\left(\tau_{n+1}-s\right)}^{\vartheta -1}\left(\left(\tau_{n}-s\right)\left(\tau_{n+1/2}-s\right)-\left(\tau_{n+1}-s\right)\left(\tau_{n}-s\right)\right)f\left(x\left(\tau_{n+1}\right),\tau_{n+1}\right)ds\right]. \end{array}$$

Evaluating all the integrals given in equation (30), we obtain

(31) $$\begin{array}{c} {\;}^{\text{ABC}}I^{\vartheta }f\left(x\left(\tau_{n+1}\right),\tau_{n+1}\right)=\frac{\left(1-\vartheta \right)}{J\left(\vartheta \right)}f\left(x\left(\tau_{n+1}\right),\tau_{n+1}\right)+\frac{\vartheta {\left(\delta \tau \right)}^{\vartheta }}{J\left(\vartheta \right)}\overset{n+1}{\underset{i=0}{\sum }}b_{n+1,i}f\left(x\left(\tau_{i}\right),\tau_{i}\right),n=0,1,2,\cdots ,N-1, \end{array}$$

where

(32) $$\begin{array}{c} b_{n+1,i}=\frac{1}{\Gamma \left(\vartheta +3\right)}\left\{\begin{array}{cc} \left(\vartheta +1\right)\left(\vartheta +2\right){\left(n+1\right)}^{\vartheta }+\left(\vartheta +2\right){\left(n\right)}^{\vartheta +1}-\left(\vartheta +2\right){\left(n+1\right)}^{\vartheta +1} & i=0,\\ -2\left(\vartheta +2\right){\left(n+1-i\right)}^{\vartheta +1}+\left(\vartheta +2\right){\left(n+2-i\right)}^{\vartheta +1}+\left(\vartheta +2\right){\left(n-i\right)}^{\vartheta +1} & 1\leq i\leq n,\\ 2+\vartheta & i=n+1. \end{array}\right. \end{array}$$

Thus we can obtain the following modified fractional Simpson's 1/3 scheme for equation (22) in ABC sense:

(33) $$\begin{array}{c} x_{n+1}=x_{0}+\frac{\left(1-\vartheta \right)}{J\left(\vartheta \right)}f\left(x\left(\tau_{n+1}\right),\tau_{n+1}\right)+\frac{\vartheta {\left(\delta \tau \right)}^{\vartheta }}{J\left(\vartheta \right)}\overset{n+1}{\underset{i=0}{\sum }}b_{n+1,i}f\left(x\left(\tau_{i}\right),\tau_{i}\right),\;n=0,1,2,\cdots ,N-1. \end{array}$$

### 4.1. Convergence and Stability Analysis

The following lemmas are very important to examine the proposed scheme's convergence and stability.

**Lemma 2 .**

Assume that *g*(*t*) ∈ *C*^3^([0, *T*]), then there exist a constant *C* such that

(34) $$\begin{array}{c} \left|\frac{1}{\Gamma \left(\vartheta \right)}\int_{\tau_{o}}^{\tau_{n+1}}{\left(\tau_{n+1}-s\right)}^{\vartheta -1}g\left(s\right)ds-{\left(\delta \tau \right)}^{\vartheta }\left(\overset{n+1}{\underset{i=0}{\sum }}b_{i}g\left(\tau_{i}\right)\right)\right|\leq \frac{T^{\vartheta }C{\left(\delta \tau \right)}^{2}}{2!\Gamma \left(\vartheta +1\right)}. \end{array}$$

**Proof**

Using the Lagrange interpolation error formula, we have

(35) $$\begin{array}{c} \left|\frac{1}{\Gamma \left(\vartheta \right)}\int_{\tau_{o}}^{\tau_{n+1}}{\left(\tau_{n+1}-s\right)}^{\vartheta -1}g\left(s\right)ds-{\left(\delta \tau \right)}^{\vartheta }\left(\overset{n+1}{\underset{i=0}{\sum }}b_{i}g\left(\tau_{i}\right)\right)\right|\leq \frac{1}{2!\Gamma \left(\vartheta \right)}\overset{n}{\underset{i=0}{\sum }}\int_{\tau_{i}}^{\tau_{i+1}}{\left(\tau_{n+1}-s\right)}^{\vartheta -1}\left|g^{\prime \prime }\left(\xi_{i}\right)\left(s-\tau_{i}\right)\left(s-\tau_{i+1}\right)\right|ds\leq \frac{C{\left(\delta \tau \right)}^{2}}{2!\Gamma \left(\vartheta \right)}\int_{\tau_{0}}^{\tau_{n+1}}{\left(\tau_{n+1}-s\right)}^{\vartheta -1}ds\leq \frac{T^{\vartheta }C{\left(\delta \tau \right)}^{2}}{2!\Gamma \left(\vartheta +1\right)}. \end{array}$$

From above lemma it is clear that the truncation error of the scheme of equation (33) is *O*((*δτ*)^2^).

**Lemma 3 .**

For 0 < *ϑ* < 1, the weights *b*_*i*_, *i* = 0, 1, 2, ⋯, *n* − 2 given in equation (33) have the following order of magnitude:

(36) $$\begin{array}{c} b_{i}=O\left({\left(n-i\right)}^{\vartheta -1}\right). \end{array}$$

**Proof**

According to the definition of *b*_*i*_(*i* = 1, 2, ⋯, *n* − 2), it deduces that

(37) $$\begin{array}{c} b_{i}=\frac{{\left(n-i\right)}^{\vartheta -1}}{\Gamma \left(\vartheta +3\right)}\left[-2\left(\vartheta +2\right){\left(n-i\right)}^{2}{\left(1+\frac{1}{n-i}\right)}^{\vartheta +1}+\left(\vartheta +2\right){\left(n-i\right)}^{2}{\left(1+\frac{2}{n-i}\right)}^{\vartheta +1}+\left(\vartheta +2\right){\left(n-i\right)}^{2}\right],\\ b_{i}=\frac{\left(\vartheta +2\right){\left(n-i\right)}^{\vartheta -1}}{\Gamma \left(\vartheta +3\right)}\left[-2\left({\left(n-i\right)}^{2}+\left(\vartheta +1\right)\left(n-i\right)+\frac{\left(\vartheta +1\right)\vartheta }{2!}+\frac{\left(\vartheta +1\right)\vartheta \left(\vartheta -1\right)}{3!}\left(\frac{1}{n-i}\right)\left.+\frac{\left(\vartheta +1\right)\vartheta \left(\vartheta -1\right)\left(\vartheta -2\right)}{4!}{\left(\frac{1}{n-i}\right)}^{2}+\cdots \right)+{\left(n-i\right)}^{2}+2\left(\vartheta +1\right){\left(n-i\right)}^{2}+\vartheta \left(\vartheta +1\right)\right.+\frac{\left(\vartheta +1\right)\vartheta \left(\vartheta -1\right)}{3!}\left(\frac{2}{n-i}\right)+\frac{\left(\vartheta +1\right)\vartheta \left(\vartheta -1\right)\left(\vartheta -2\right)}{4!}{\left(\frac{2}{n-i}\right)}^{2}+\cdots +{\left(n-i\right)}^{2}\right], \end{array}$$

implies

(38) $$\begin{array}{c} b_{i}=\frac{\left(\vartheta +2\right){\left(n-i\right)}^{\vartheta -1}}{\Gamma \left(\vartheta +3\right)}\left[\frac{2\left(\vartheta +1\right)\vartheta \left(\vartheta -1\right)\left(\vartheta -2\right)}{4!}{\left(\frac{1}{n-i}\right)}^{2}+\frac{6\left(\vartheta +1\right)\vartheta \left(\vartheta -1\right)\left(\vartheta -2\right)\left(\vartheta -3\right)}{5!}{\left(\frac{1}{n-i}\right)}^{3}\right.\left.+\frac{14\left(\vartheta +1\right)\vartheta \left(\vartheta -1\right)\left(\vartheta -2\right)\left(\vartheta -3\right)\left(\vartheta -4\right)}{6!}{\left(\frac{1}{n-i}\right)}^{4}+\cdots \right]. \end{array}$$

Note that 0 < *ϑ* < 1, so the coefficients of power of 1/(*n* − *i*) are less than 1. Thus, the series given above is convergent, and hence the proof is completed for *b*_*i*_(*i* = 1, 2, ⋯, *n* − 2). Similar strategy can be adopted for *b*_*n*_, so we neglect the proof.

**Theorem 2 .**

The numerical scheme (33) is conditionally convergent. That is, for 0 < *ϑ* ≤ 1 and a sufficiently small *δτ*, there exist a constant *C*_1_ such that

(39) $$\begin{array}{c} \left\|x\left(\tau_{n+1}\right)-x_{n+1}\right\|\leq C_{1}\delta \tau^{2}. \end{array}$$

**Proof**

To prove the theorem, considering the difference between actual solution and approximate solution, we get

(40) $$\begin{array}{c} x\left(\tau_{n+1}\right)-x_{n+1}=\frac{\left(1-\vartheta \right)}{J\left(\vartheta \right)}\left[f\left(x\left(\tau_{n+1}\right),\tau_{n+1}\right)-f\left(x_{n+1},\tau_{n+1}\right)\right]+\frac{\vartheta }{J\left(\vartheta \right)\Gamma \left(\vartheta \right)}\int_{0}^{\tau_{n+1}}{\left(\tau_{n+1}-s\right)}^{\vartheta -1}f\left(x\left(s\right),s\right)ds-\frac{\vartheta {\left(\delta \tau \right)}^{\vartheta }}{J\left(\vartheta \right)}\overset{n+1}{\underset{i=0}{\sum }}b_{n+1,i}f\left(x_{i},\tau_{i}\right)=\frac{\left(1-\vartheta \right)}{J\left(\vartheta \right)}\left[f\left(x\left(\tau_{n+1}\right),\tau_{n+1}\right)-f\left(x_{n+1},\tau_{n+1}\right)\right]+\frac{\vartheta {\left(\delta \tau \right)}^{\vartheta }}{J\left(\vartheta \right)}\overset{n+1}{\underset{i=0}{\sum }}b_{n+1,i}\left(f\left(x\left(\tau_{i}\right),\tau_{i}\right)-f\left(x_{i},\tau_{i}\right)\right)+\frac{\vartheta }{J\left(\vartheta \right)}\left[\frac{1}{\Gamma \left(\vartheta \right)}\int_{0}^{\tau_{n+1}}{\left(\tau_{n+1}-s\right)}^{\vartheta -1}f\left(x\left(s\right),s\right)ds-{\left(\delta \tau \right)}^{\vartheta }\overset{n+1}{\underset{i=0}{\sum }}b_{n+1,i}f\left(x\left(\tau_{i}\right),\tau_{i}\right)\right],\\ \left\|x\left(\tau_{n+1}\right)-x_{n+1}\right\|=\left\|\frac{\left(1-\vartheta \right)}{J\left(\vartheta \right)}\left[f\left(x\left(\tau_{n+1}\right),\tau_{n+1}\right)-f\left(x_{n+1},\tau_{n+1}\right)\right]+\frac{\vartheta {\left(\delta \tau \right)}^{\vartheta }}{J\left(\vartheta \right)}\overset{n+1}{\underset{i=0}{\sum }}\left(f\left(x\left(\tau_{i}\right),\tau_{i}\right)-f\left(x_{i},\tau_{i}\right)\right)\right\|+\frac{\vartheta }{J\left(\vartheta \right)}\left[\frac{1}{\Gamma \left(\vartheta \right)}\int_{0}^{\tau_{n+1}}{\left(\tau_{n+1}-s\right)}^{\vartheta -1}f\left(x\left(s\right),s\right)ds-{\left(\delta \tau \right)}^{\vartheta }\overset{n+1}{\underset{i=0}{\sum }}b_{n+1,i}f\left(x\left(\tau_{i}\right),\tau_{i}\right)\right]. \end{array}$$

Using Lipschitz condition of equation (23) after applying triangle inequality and using Lemma 4.1, we get

(41) $$\begin{array}{c} \left\|x\left(\tau_{n+1}\right)-x_{n+1}\right\|\leq \frac{\left(1-\vartheta \right)}{J\left(\vartheta \right)}\left\|f\left(x\left(\tau_{n+1}\right),\tau_{n+1}\right)-f\left(x_{n+1},\tau_{n+1}\right)\right\|+\frac{\vartheta {\left(\delta \tau \right)}^{\vartheta }}{J\left(\vartheta \right)}\overset{n+1}{\underset{i=0}{\sum }}b_{n+1,i}\left\|f\left(x\left(\tau_{i}\right),\tau_{i}\right)-f\left(x_{i},\tau_{i}\right)\right\|+\frac{\vartheta }{J\left(\vartheta \right)}\left\|\frac{1}{\Gamma \left(\vartheta \right)}\int_{0}^{\tau_{n+1}}{\left(\tau_{n+1}-s\right)}^{\vartheta -1}f\left(x\left(s\right),s\right)ds-{\left(\delta \tau \right)}^{\vartheta }\overset{n+1}{\underset{i=0}{\sum }}b_{n+1,i}f\left(x\left(\tau_{i}\right),\tau_{i}\right)\right\|\leq \frac{\left(1-\vartheta \right)L}{J\left(\vartheta \right)}\left\|x\left(\tau_{n+1}\right)-x_{n+1}\right\|+\frac{\vartheta T^{\vartheta }}{J\left(\vartheta \right)}\frac{C{\left(\delta \tau \right)}^{2}}{2\Gamma \left(\vartheta +1\right)}+\frac{\vartheta {\left(\delta \tau \right)}^{\vartheta }L}{J\left(\vartheta \right)}\overset{n+1}{\underset{i=0}{\sum }}b_{n+1,i}\left\|x\left(\tau_{i}\right)-x_{i}\right\|\leq \frac{L}{J\left(\vartheta \right)}\left(1-\vartheta +\frac{\vartheta {\left(\delta \tau \right)}^{\vartheta }}{\Gamma \left(\vartheta +3\right)}\right)\left\|x\left(\tau_{n+1}\right)-x_{n+1}\right\|+\frac{\vartheta T^{\vartheta }}{J\left(\vartheta \right)}\frac{C{\left(\delta \tau \right)}^{2}}{2\Gamma \left(\vartheta +1\right)}+\frac{\vartheta {\left(\delta \tau \right)}^{\vartheta }L}{J\left(\vartheta \right)}\overset{n}{\underset{i=0}{\sum }}b_{n+1,i}\left\|x\left(\tau_{i}\right)-x_{i}\right\|. \end{array}$$

Now using Lemma 4.2 under the condition (*L*/*J*(*ϑ*))(1 − *ϑ* + (*ϑδτ*^*ϑ*^/Γ(*ϑ* + 3))) < 1, we get

(42) $$\begin{array}{c} \left\|x\left(\tau_{n+1}\right)-x_{n+1}\right\|\leq g\left(\delta \tau ,\vartheta \right)\frac{\vartheta T^{\vartheta }}{J\left(\vartheta \right)}\frac{C{\left(\delta \tau \right)}^{2}}{2\Gamma \left(\vartheta +1\right)}+g\left(\delta \tau ,\vartheta \right)\frac{\vartheta {\left(\delta \tau \right)}^{\vartheta }L}{J\left(\vartheta \right)}\overset{n}{\underset{i=0}{\sum }}{\left(n-i\right)}^{\vartheta -1}\left\|x\left(\tau_{i}\right)-x_{i}\right\|, \end{array}$$

where *g*(*δτ*, *ϑ*) = (*J*(*ϑ*)Γ(*ϑ* + 3))/(*J*(*ϑ*)Γ(*ϑ* + 3) − *L*((Γ(*ϑ* + 3)(1 − *ϑ*) + *ϑδτ*^*ϑ*^)) For any 0 < *ϑ* < 1 and a sufficiently small *δτ*, there exist a constant *C*_*g*_ such that

(43) $$\begin{array}{c} 1<g\left(\delta \tau ,\vartheta \right)<C_{g}. \end{array}$$

Hence by applying Gronwall inequality given in Lemma 2.1 and using the property (43), we conclude

(44) $$\begin{array}{c} \left\|x\left(\tau_{n+1}\right)-x_{n+1}\right\|\leq C_{1}\delta \tau^{2}. \end{array}$$

**Theorem 3 .**

For 0 < *ϑ* ≤ 1 and a sufficiently small *δτ*, there exist a constant *C*_1_ such that the numerical scheme (33) is stable.

**Proof**

To prove the theorem, let the perturbation of *x*_*n*_ and *x*_0_ be denoted by ${\tilde{x}}_{n}$ and ${\tilde{x}}_{0}$, respectively, for *n* = 0, 1, ⋯, *N* − 1. Adding this perturbation to the numerical scheme (33) we get

(45) $$\begin{array}{c} x_{n+1}+{\tilde{x}}_{n+1}=x_{0}+{\tilde{x}}_{0}+\frac{\left(1-\vartheta \right)}{J\left(\vartheta \right)}f\left(x_{n+1}+{\tilde{x}}_{n+1}\right)+\frac{\vartheta {\left(\delta \tau \right)}^{\vartheta }}{J\left(\vartheta \right)}\overset{n+1}{\underset{i=0}{\sum }}b_{n+1,i}f\left(x_{i}+{\tilde{x}}_{i}\right). \end{array}$$

Subtracting equation (33) from equation (45), we get

(46) $$\begin{array}{c} {\tilde{x}}_{n+1}={\tilde{x}}_{0}+\frac{\left(1-\vartheta \right)}{J\left(\vartheta \right)}\left[f\left(x_{n+1}+{\tilde{x}}_{n+1}\right)-f\left(x_{n+1}\right)\right]+\frac{\vartheta {\left(\delta \tau \right)}^{\vartheta }}{J\left(\vartheta \right)}\overset{n+1}{\underset{i=0}{\sum }}b_{n+1,i}\left(f\left(x_{i}+{\tilde{x}}_{i}\right)-f\left(x_{i}\right)\right). \end{array}$$

Using the Lipschitz condition followed by triangle inequality, we get

(47) $$\begin{array}{c} \left\|{\tilde{x}}_{n+1}\right\|=\left\|{\tilde{x}}_{0}+\frac{\left(1-\vartheta \right)}{J\left(\vartheta \right)}\left[f\left(x_{n+1}+{\tilde{x}}_{n+1}\right)-f\left(x_{n+1}\right)\right]+\frac{\vartheta {\left(\delta \tau \right)}^{\vartheta }}{J\left(\vartheta \right)}\overset{n+1}{\underset{i=0}{\sum }}b_{n+1,i}\left(f\left(x_{i}+{\tilde{x}}_{i}\right)-f\left(x_{i}\right)\right)\right\|,\leq \left\|{\tilde{x}}_{0}\right\|+\frac{\left(1-\vartheta \right)}{J\left(\vartheta \right)}\left\|f\left(x_{n+1}+{\tilde{x}}_{n+1}\right)-f\left(x_{n+1}\right)\right\|+\frac{\vartheta {\left(\delta \tau \right)}^{\vartheta }}{J\left(\vartheta \right)}\overset{n+1}{\underset{i=0}{\sum }}b_{n+1,i}\left\|f\left(x_{i}+{\tilde{x}}_{i}\right)-f\left(x_{i}\right)\right\|,\leq \left\|{\tilde{x}}_{0}\right\|+\frac{\left(1-\vartheta \right)L}{J\left(\vartheta \right)}\left\|{\tilde{x}}_{n+1}\right\|+\frac{\vartheta {\left(\delta \tau \right)}^{\vartheta }L}{J\left(\vartheta \right)}\overset{n+1}{\underset{i=0}{\sum }}b_{n+1,i}\left\|{\tilde{x}}_{i}\right\|,\leq \left\|{\tilde{x}}_{0}\right\|+\frac{L}{J\left(\vartheta \right)}\left(1-\vartheta +\frac{\vartheta {\left(\delta \tau \right)}^{\vartheta }}{\Gamma \left(\vartheta +3\right)}\right)\left\|{\tilde{x}}_{n+1}\right\|+\frac{\vartheta {\left(\delta \tau \right)}^{\vartheta }L}{J\left(\vartheta \right)}\overset{n}{\underset{i=0}{\sum }}b_{n+1,i}\left\|{\tilde{x}}_{i}\right\|. \end{array}$$

Now if (*L*/*J*(*ϑ*))(1 − *ϑ* + (*ϑδτ*^*ϑ*^/Γ(*ϑ* + 3))) < 1, then using Lemma 4.2 we get

(48) $$\begin{array}{c} \left\|{\tilde{x}}_{n+1}\right\|\leq g\left(\delta \tau ,\vartheta \right)\left\|{\tilde{x}}_{0}\right\|+g\left(\delta \tau ,\vartheta \right)\frac{\vartheta \delta \tau^{\vartheta }L}{J\left(\vartheta \right)}\overset{n}{\underset{i=0}{\sum }}{\left(n-i\right)}^{\vartheta -1}\left\|{\tilde{x}}_{i}\right\|, \end{array}$$

where *g*(*δτ*, *ϑ*) = *J*(*ϑ*)Γ(*ϑ* + 3)/(*J*(*ϑ*)Γ(*ϑ* + 3) − *L*(Γ(*ϑ* + 3)(1 − *ϑ*) + *ϑδτ*^*ϑ*^).

Using property (43), we have

(49) $$\begin{array}{c} \left\|{\tilde{x}}_{n+1}\right\|\leq C_{g}\left\|{\tilde{x}}_{0}\right\|+C_{g}\frac{\vartheta {\left(\delta \tau \right)}^{\vartheta }L}{J\left(\vartheta \right)}\overset{n}{\underset{i=0}{\sum }}{\left(n-i\right)}^{\vartheta -1}\left\|{\tilde{x}}_{i}\right\|. \end{array}$$

Hence by applying the Gronwall inequality given in Lemma 2.1, we conclude

(50) $$\begin{array}{c} \left\|{\tilde{x}}_{n+1}\right\|\leq C_{1}\left\|{\tilde{x}}_{0}\right\|. \end{array}$$

## 5. Fractional Model

Employing Atangana-Baleanu fractional order derivative in Caputo sense of order *ϑ* on system of equation (7), we have the following fractional model,

(51) DABCτϑSτ=Λ−μS−δS−βSIN,ABCDτϑEτ=βSIN−μ+εE+σβVIN,ABCDτϑIτ=εE−γ+μ+ϑI,ABCDτϑRτ=γI−μR,ABCDτϑVτ=δS−μV−σβVIN,

along with initial conditions

(52) $$\begin{array}{c} S\left(0\right)=S_{0},E\left(0\right)=E_{0},I\left(0\right)=I_{0},R\left(0\right)=R_{0},V\left(0\right)=V_{0}. \end{array}$$

Adopting the previously defined procedure, model of equation (51) takes the form

(53) DABCτϑSτ=X1t,S,E,I,R,V,ABCDτϑEτ=X2t,S,E,I,R,V,DABCτϑIτ=X3t,S,E,I,R,V,DABCτϑRτ=X4t,S,E,I,R,V,DABCτϑVτ=X5t,S,E,I,R,V.

Furthermore applying the numerical scheme(33), system (53) becomes

(54) $$\begin{array}{c} S\left(\tau_{n+1}\right)=S_{0}+\frac{\left(1-\vartheta \right)}{J\left(\vartheta \right)}X_{1}\left(\tau ,S,E,I,R,V\right)+\frac{\vartheta {\left(\delta \tau \right)}^{\vartheta }}{J\left(\vartheta \right)}\overset{n+1}{\underset{i=0}{\sum }}b_{n+1,i}X_{1}\left(\tau ,S,E,I,R,V\right),\\ E\left(\tau_{n+1}\right)=E_{0}+\frac{\left(1-\vartheta \right)}{J\left(\vartheta \right)}X_{2}\left(\tau ,S,E,I,R,V\right)+\frac{\vartheta {\left(\delta \tau \right)}^{\vartheta }}{J\left(\vartheta \right)}\overset{n+1}{\underset{i=0}{\sum }}b_{n+1,i}X_{2}\left(\tau ,S,E,I,R,V\right),\\ I\left(\tau_{n+1}\right)=I_{0}+\frac{\left(1-\vartheta \right)}{J\left(\vartheta \right)}X_{3}\left(\tau ,S,E,I,R,V\right)+\frac{\vartheta {\left(\delta \tau \right)}^{\vartheta }}{J\left(\vartheta \right)}\overset{n+1}{\underset{i=0}{\sum }}b_{n+1,i}X_{3}\left(\tau ,S,E,I,R,V\right),\\ R\left(\tau_{n+1}\right)=R_{0}+\frac{\left(1-\vartheta \right)}{J\left(\vartheta \right)}X_{4}\left(\tau ,S,E,I,R,V\right)+\frac{\vartheta {\left(\delta \tau \right)}^{\vartheta }}{J\left(\vartheta \right)}\overset{n+1}{\underset{i=0}{\sum }}b_{n+1,i}X_{4}\left(\tau ,S,E,I,R,V\right),\\ V_{0}+\frac{\left(1-\vartheta \right)}{J\left(\vartheta \right)}X_{5}\left(\tau ,S,E,I,R,V\right)+\frac{\vartheta {\left(\delta \tau \right)}^{\vartheta }}{J\left(\vartheta \right)}\overset{n+1}{\underset{i=0}{\sum }}b_{n+1,i}X_{5}\left(\tau ,S,E,I,R,V\right), \end{array}$$

where *a*_*n*+1,*k*_ are already defined.

### 5.1. The Positivity and Boundness of the Solution

In this subsection we will discuss the positive nature of the epidemiological model of equation (51). We will recall the following lemma for the proof of the main theorem on the positivity of the solution of the fractional model (51).

**Lemma 4 .**

Generalized Mean Value Theorem: let *ϕ*(*τ*) ∈ *C*[*a*, *b*] and Atangana-Baleanu fractional order derivative, ^ABC^*D*_*τ*_^*ϑ*^*ϕ*(*τ*) ∈ *C*(*a*, *b*]*for*0 < *ϑ* ≤ 1, then

(55) $$\begin{array}{c} \phi \left(\tau \right)=\phi \left(s\right)+{\frac{1-\vartheta }{J\left(\vartheta \right)}}^{\text{ABC}}D^{\vartheta }\phi \left(\tau \right)+{\frac{1}{J\left(\vartheta \right)\Gamma \left(\vartheta \right)}}^{\text{ABC}}D^{\vartheta }\phi \left(u\right){\left(\tau -s\right)}^{\vartheta } \end{array}$$

with 0 ≤ *u* ≤ *τ*, ∀*τ* ∈ (*a*, *b*].

**Remark 1 .**

Let *ϕ*(*τ*) ∈ *C*[0, *b*] and Atangana-Baleanu fractional order derivative, ^ABC^*D*_*τ*_^*ϑ*^ ∈ (0, *b*) for 0 < *ϑ* ≤ 1.  Lemma 5.1 shows that if  ^ABC^*D*_*τ*_^*ϑ*^*ϕ*(*τ*) > 0∀ *τ* ∈ (0, *b*], then the function *ϕ*(*τ*) is nondecreasing and if  ^ABC^*D*_*τ*_^*ϑ*^*ϕ*(*τ*) ≤ 0∀ *τ* ∈ (0, *b*] then *ϕ*(*τ*) is nonincreasing for all *τ* ∈ [0, *b*].

**Theorem 4 .**

The solution to the nonnegative initial conditions of equation (52) of the proposed model of equation (51) is unique and limited in *R*_+_^5^.

**Proof**

The existence and uniqueness of the model solution of equations (51) and (52) can be achieved in the time interval (0, ∞) by [35]. The nonnegative region *R*_+_^5^ would seem to be a positive invariant region that must be represented. We observe from the model of equation (51)

(56) $$\begin{array}{c} \begin{array}{c} {}^{\text{ABC}}D_{\tau }^{\vartheta }S\left(\tau \right)\left|{}_{S=0}\right.=\Lambda ,\\ {}^{\text{ABC}}D_{\tau }^{\vartheta }E\left(\tau \right)\left|{}_{E=0}\right.=\beta S\frac{I}{N}+\sigma \beta V\frac{I}{N},\\ {}^{\text{ABC}}D_{\tau }^{\vartheta }I\left(\tau \right)\left|{}_{I=0}\right.=\in E,\\ {}^{\text{ABC}}D_{\tau }^{\vartheta }R\left(\tau \right)\left|{}_{R=0}\right.=\gamma I,\\ {}^{\text{ABC}}D_{\tau }^{\vartheta }V\left(\tau \right)\left|{}_{V=0}\right.=\delta S. \end{array} \end{array}$$

From Remark 1 and system of equation (56), the solution (*S*(0), *E*(0), *I*(0), *R*(0), *V*(0)) ∈ *R*_+_^5^. Also, in each line bounded the nonnegative octant, the vector field points will remain in *R*_+_^5^. Therefore, the fractional model of equation (51) of a solution ((*S*(*τ*), *E*(*τ*), *I*(*τ*), *R*(*τ*), *V*(*τ*)) is nonnegative if the initial condition is set positively to invariant.

## 6. Numerical Results and Discussion

Considering the case of Italy, we applied the proposed model to analyse the impact of vaccination. The vaccination campaign for *COVID-19* started on 27^th^ December 2020 in Italy managed by the Ministry of Health. In the early months of the vaccination campaign, the Italian government targeted health doctors and administrative staff as well as guests and nursing home personnel followed the vaccination of elderly people and public service personnel in second phase of the campaign. Italian government bought four out of seven, WHO approved vaccines to facilitate its people against the virus. So far, 73.3% of the total population has received at least one dose and 65.5% of the total population is fully vaccinated. As of 17^*th*^ September 2021, top ten regions of Italy for the total number of administered *COVID-19* vaccine doses can be seen in Figure 2. Moreover the number of people who received at least one dose and fully vaccinated according to the data [19] are presented in Figure 3.

Further, graphical presentation of the numerical simulation for the fractional model (51) are given in this section.  Table 1 shows the estimated model parameters and initial values used to evaluate the impact of vaccination on the *COVID-19* epidemic.

Figure 4 shows the impact by varying the vaccination rates on different classes of the proposed model with *δ* = 0 representing the model output without vaccination. Although there is no remarkable change in the graph of susceptible class, we can observe a significant decrease in infected and exposed classes by increasing the vaccination rate. We can see the peak of the infected as well as that of exposed individuals gradually decreases with the increase in effective rate of vaccination. From Figure 4, we can observe that for exposed class there is a difference of almost 7 × 10^6^ individuals in peak values for no vaccination to a vaccination rate *δ* = 0.012. Similarly, the peak values for no vaccination compared to a vaccination rate of *δ* = 0.012 for the infected class differ by almost 7 × 10^6^ individuals. So, interpreting graphically the dynamics of the proposed model to observe the effect of vaccination by altering the vaccination rate suggest that, mass vaccination along with the implementation of the control measures until the achievement of complete herd immunity is needed to control the spread of the disease. Hence, majority of susceptible population should be vaccinated to prevent the new waves of COVID-19. The vaccination of the susceptible class will control the spread of the disease resulting in reduction of the mortality rate, which can clearly be seen by recovered class presented in Figure 4. Simulation results show that immunization is an essential strategy for lowering the incidence and severity of *COVID-19* infections in the workplace, in communities, and across the globe. Therefore, it is advocated for policymakers to increase public trust and confidence in the efficiency and security of vaccinations as well as the expertise and dependability of the institutions that provide them. Figures 5 and 6 show a comparison of integer order model, fractional model for fractional order *ϑ* = 0.975,0.95,0.925, 0.9, and real data of total number of deaths *D* = *ϑI* owing to the *COVID-19* outbreak in Italy.  Figure 5 presents the comparison for first 80 days starting from 23^*rd*^ February 2020 to 13^*th*^ May 2020 of the pandemic before vaccination. We can see that after 40 days, real data is better explained by fractional order model in comparison to integer order.  Figure 6 is assigned to display the comparison from 1^*st*^ July 2021 to 19^*th*^ September 2021 along with administered vaccination effect considering the initial values of the compartments as of 1^*st*^ July 2021 . The relevant *COVID-19* data can be found at https://github.com/pcmdpc/COVID-19. Also we can see from our proposed model, fractional order models are better at fitting the real data than classical models because fractional order derivative and integral operators, due to their nonlocal nature, depend not only on their current state but also on all of their previous states, making them more effective than other classical deterministic operators in predicting the biological model's future state.

## 7. Concluding Remarks

Within the Atangana-Baleanu Caputo fractional operator, we studied alternative conditions for qualitative characterization and dynamics of the suggested model. Calculating disease-free and endemic equilibrium points, as well as the reproduction number, are used to examine the prerequisites for local stability. A newly developed numerical scheme is used to obtain the solution of the concerned fractional order model. The proposed scheme's stability and convergence are briefly examined. To depict the behaviour of the *COVID-19* virus, a graphical description of the dynamics of the relevant system is developed within different fractional orders under the effect of vaccination suggesting the need of mass vaccination to gain the herd immunity in order to prevent the further spread of the disease. Due to the limited access of the available vaccine, other preventive measures should also be continued.

## Figures and Tables

**Figure 1:** SEIRV Model.

**Figure 2:** Number of *COVID-19* vaccine doses administered in Italy (top ten regions).

**Figure 3:** Number of Vaccinated People.

**Figure 4:** Impact of vaccination rate on all the four susceptible, exposed, infected, and recovered classes.

**Figure 5:** Comparison of the number of people who died for various fractional orders vs. real data (before vaccination).

**Figure 6:** Comparison of the number of people who died for various fractional orders vs. real data (after vaccination).

**Table 1:** Parameter and initial values for the numerical simulations.

Parameter	Value	Parameter	Value	Initial time model variables	Value
N	60000000	*ε*	1/4.02	*S*(0)	59988539
*μ*	0.0000373	*Λ*	*μ* × *N*	*E*(0)	11460
*γ*	1/5.25	*ϑ*	0.00144	*I*(0)	1
*β*	0.75	*σ*	0.25	*R*(0)	0

## Data Availability

The data used to support the findings of this study can be found at https://ourworldindata.org/covid-vaccinations.

## References

[1] Zhang Z. (2020). A novel covid-19 mathematical model with fractional derivatives: singular and nonsingular kernels. *Chaos, Solitons and Fractals*.

[2] Rezapour S., Mohammadi H., Samei M. E. (2020). SEIR epidemic model for COVID-19 transmission by Caputo derivative of fractional order. *Advances in Difference Equations*.

[3] Atangana A., İğret A. S. (2020). Mathematical model of COVID-19 spread in Turkey and South Africa: theory, methods, and applications. *Advances in Difference Equations*.

[4] Zhang Z., Zeb A., Egbelowo O. F., Erturk V. S. (2020). Dynamics of a fractional order mathematical model for COVID-19 epidemic. *Adv. Difference Equ.*.

[5] Ahmad S., Aman Ullah Q. M., Al-Mdallal H., Khan K., Shah A. K. (2020). Fractional order mathematical modeling of COVID-19 transmission. *Chaos, Solitons and Fractals*.

[6] Zakary O., Bidah S., Rachik M., Ferjouchia H. (2020). Mathematical model to estimate and predict the covid-19 infections in morocco: optimal control strategy. *Journal of Applied mathematics*.

[7] Ahmad Z., Arif M., Ali F., Khan I., Nisar K. S. (2020). A report on COVIDâ€‘19 epidemic in pakistan using SEIR fractional model. *Scientific Reports*.

[8] Askar S. S., Ghosh D., Santra P. K., Abdelalim A., Elsadany G. S. M. (2021). A fractional order SITR mathematical model for forecasting of transmission of COVID-19 of India with lockdown effect. *Results in Physics*.

[9] Bushnaq S., Saeed T., Torres D. F. M., Zeb A. (2021). Control of COVID-19 dynamics through a fractional-order model. *Alexandria Engineering Journal*.

[10] Abdulwasaa M. A., Abdo M. S., Shah K. (2021). Fractal-fractional mathematical modeling and forecasting of new cases and deaths of COVID-19 epidemic outbreaks in India. *Results in Physics*.

[11] Baba I. A., Rihan A. (2022). A fractional-order model with different strains of COVID-19. *Physica A*.

[12] Rihan F. A., Gandhi V. (2021). Dynamics and sensitivity of fractional-oder delay differential model for coronavirus (COVID-19) infection. *Progress in Fractional Differentiation and Applications*.

[13] Rihan F. A., Alsakaji H. J. (2021). Dynamics of a stochastic delay differential model for COVID-19 infection with asymptomatic infected and interacting people: case study in the UAE. *Results in Physics*.

[14] Furati K. M., Sarumi I. O., Khaliq A. Q. M. (2021). Fractional model for the spread of COVID-19 subject to government intervention and public perception. *Applied Mathematical Modelling*.

[15] Alqahtani R. T. (2021). Mathematical model of SIR epidemic system (COVID-19) with fractional derivative: stability and numerical analysis. *Advances in Difference Equations*.

[16] Hattaf K. (2020). A new generalized definition of fractional derivative with non-singular kernel. *Computation*.

[17] Hattaf K. (2022). On the stability and numerical scheme of fractional differential equations with application to biology. *Computation*.

[18] Regassa Cheneke K., Purnachandra Rao K., Kenassa E. G. (2022). A new generalized fractional-order derivative and bifurcation analysis of cholera and human immunodeficiency co-infection dynamic transmission. *International Journal of Mathematics and Mathematical Sciences*.

[19] https://ourworldindata.org/covid-vaccinations.

[20] Meng X., Cai Z., Si S., Duan D. (2021). Analysis of epidemic vaccination strategies on heterogeneous networks: based on SEIRV model and evolutionary game. *Applied Mathematics and Computation*.

[21] Ramos A. M., Vela-Pérez M., Ferrández M. R., Kubik A. B., Ivorra B. (2021). Modeling the impact of SARS-CoV-2 variants and vaccines on the spread of COVID-19. *Communications in Nonlinear Science and Numerical Simulation*.

[22] Tetteh J. N. A., Nguyen V. K., Hernandez-Vargas E. A. (2020). COVID-19 network model to evaluate vaccine strategies towards herd immunity. https://www.medrxiv.org/content/10.1101/2020.12.22.20248693v1.

[23] Harizi I., Berkan S., Tayebi A. (2020). Modeling the effect of population-wide vaccination on the evolution of COVID-19 epidemic in Canada. https://www.medrxiv.org/content/10.1101/2021.02.05.21250572v2.

[24] Karabay A., Kuzdeuov A., Lewis M., Varo H. A. (2021). A vaccination simulator for COVID-19: effective and sterilizing immunization cases. https://www.medrxiv.org/content/10.1101/2021.03.28.21254468v2.

[25] Tuteja G. S. (2020). Stability and numerical investigation of modified SEIR model with vaccination and life-long immunity. *European Journal of Molecular and Clinical Medicine.*.

[26] Ghostine R., Gharamti M., Hassrouny S., Hoteit I. (2021). An extended SEIR model with vaccination for forecasting the COVID-19 pandemic in Saudi Arabia using an ensemble Kalman filter. *Mathematics*.

[27] Wintachaia P., Prathomb K. (2021). Stability analysis of SEIR model related to efficiency of vaccines for COVID-19 situation. *Heliyon*.

[28] Alsakaji H. J., Rihan F. A., Hashish A. (2022). Dynamics of a stochastic epidemic model with vaccination and multiple time- delays for COVID-19 in the UAE. *Complexity*.

[29] Kou L., Wang X., Li Y., Guo X., Zhang H. (2021). A multi-scale agent-based model of infectious disease transmission to assess the impact of vaccination and non-pharmaceutical interventions: the COVID-19 case. *Journal of Safety Science and Resilience*.

[30] Acuña-Zegarra M. A., Díaz-Infante S., Baca-Carrasco D., Olmos-Liceaga D. (2021). COVID-19 optimal vaccination policies: a modeling study on efficacy, natural and vaccine-induced immunity responses. *Mathematical Biosciences*.

[31] Albani V. V., Loria J., Massad E., Zubelli J. P. (2021). The impact of COVID-19 vaccination delay: a data-driven modeling analysis for Chicago and New York City. *Vaccine*.

[32] Atangana A., Baleanu D. (2016). New fractional derivatives with nonlocal and non-singular kernel: theory and application to heat transfer model. *Thermal Science*.

[33] Huang J., Yang D. (2017). A unified difference-spectral method for time-space fractional diffusion equations. *International Journal of Computer Mathematics*.

[34] Van den Driessche P., Watmough J. (2002). Reproduction numbers and sub-threshold endemic equilibria for compartmental models of disease transmission. *Mathematical Biosciences*.

[35] Lin W. (2007). Global existence theory and chaos control of fractional differential equations. *Journal of Mathematical Analysis and Applications*.

